The article "Curcumin Improves Palmitate-Induced Insulin Resistance in Human Umbilical Vein Endothelial Cells by Maintaining Proteostasis in Endoplasmic Reticulum" was retracted in 2023. Reasons: original data or images not available; unreliable data; unreliable results or conclusions; concerns about the images.

# Curcumin Improves Palmitate-Induced Insulin Resistance in Human Umbilical Vein Endothelial Cells by Maintaining Proteostasis in Endoplasmic Reticulum

**DOI:** 10.3389/fphar.2017.00148

**Published:** 2017-03-21

**Authors:** Mao Ye, Hong Qiu, Yingkang Cao, Min Zhang, Yan Mi, Jing Yu, Changhua Wang

**Affiliations:** ^1^Department of Endocrinology, The Central Hospital of Enshi Autonomous PrefectureEnshi, China; ^2^Department of Pathology and Pathophysiology, School of Basic Medical Sciences, Wuhan UniversityWuhan, China; ^3^Department of Laboratory, Dongfeng General Hospital of Hubei Medical UniversityShiyan, China

**Keywords:** curcumin, insulin resistance, endoplasmic reticulum stress, autophagy, ubiquitin-proteasome system, human umbilical vein endothelial cells

## Abstract

Dysfunction of proteasome and autophagy will result in disturbance of endoplasmic reticulum (ER) proteostasis, and thus lead to long-term and chronic ER stress and subsequent unfolded protein response (UPR), which is implicated in the occurrence and development of insulin resistance. Curcumin exerts beneficial metabolic effects in *in vitro* cells and *in vivo* animal models of diabetes and diabetic complications including cardiovascular diseases, due to its powerful anti-oxidative and anti-inflammatory properties. However, its impacts on insulin resistance of endothelial cells and its underlying mechanism(s) remain ill-defined. Herein, we tested the hypothesis that curcumin action in ER protein quality control was related to improvement of insulin resistance in human umbilical vein endothelial cells (HUVECs) cultured with saturated fatty acid palmitate. We found that palmitate treatment induced insulin resistance of HUVECs and activated both the ubiquitin-proteasome system (UPS) and autophagy. Palmitate-stimulated activation of the UPS and autophagy was attenuated by pharmacological inhibition of ER stress. In addition, curcumin supplementation mitigated palmitate-induced insulin resistance, inhibited the UPS, and activated autophagy. Furthermore, curcumin administration suppressed palmitate-induced protein aggregation and ER stress. Genetic inhibition of autophagy by silencing autophagy protein 5 (Atg5) completely restored total protein ubiquitination and protein aggregation in HUVECs treated with combined curcumin and palmitate. Atg5-knockdown also abolished the beneficial effects of curcumin on palmitate-induced ER stress, JNK/IRS-1 pathway as well as insulin signaling. Our results reveal that curcumin-activated autophagy could maintain proteostasis in ER leading to attenuation of ER stress and subsequent inhibition of JNK/IRS-1 pathway and improvement of insulin resistance.

The article "Curcumin Improves Palmitate-Induced Insulin Resistance in Human Umbilical Vein Endothelial Cells by Maintaining Proteostasis in Endoplasmic Reticulum" was retracted in 2023. Reasons: original data or images not available; unreliable data; unreliable results or conclusions; concerns about the images.

## Introduction

Endothelial dysfunction plays a critical role in the development of diabetic complications including diabetic cardiovascular disorders (Hadi and Suwaidi, 2007; Leucker and Jones, 2014; Tang et al., 2014; Dhananjayan et al., 2016). A growing body of evidence suggests that abnormality of vascular endothelium can be individually or collectively promoted by various risk factors occurred in diabetes such as oxidative stress, inflammation, hyperglycemia, and hyperlipidemia (Prieto et al., 2014; Dhananjayan et al., 2016; Riehle and Abel, 2016). Insulin resistance closely associated with the pathogenesis of diabetes and early heart diseases has also been implicated in endothelial dysfunction (Prieto et al., 2014; Janus et al., 2016). Importantly, insulin resistance and endothelial dysfunction appear to affect each other by several signaling pathways and precede the development of overt hyperglycemia in diabetic individuals (Hadi and Suwaidi, 2007; Bertoluci et al., 2015; Janus et al., 2016). Therefore, targeting insulin resistance of vascular endothelial cells may bring to bear beneficial metabolic effects for preventing the diabetic-related cardiovascular diseases.

Curcumin, a major bioactive component from ancient medicinal herb *Curcuma longa* L., has shown strong ability to improve diabetes and diabetic complications, due to its physiological and pharmacological properties such as anti-oxidative stress, anti-inflammation, and anti-insulin resistance activities (Jeenger et al., 2015; Nabavi et al., 2015; Rivera-Mancía et al., 2015). Numerous *in vitro* and *in vivo* studies have documented that curcumin sensitizes insulin action or activates insulin signaling under various pathological and pathophysiological conditions (Chuengsamarn et al., 2012; Shao et al., 2012; Wang et al., 2016; Weisberg et al., 2016). In contrast, high concentration of curcumin has been reported to directly or indirectly inhibit insulin signaling pathway and glucose transport in 3T3-L1 adipocytes under normal culture condition (Ikonomov et al., 2002; Green et al., 2014; Zhang et al., 2016). These studies suggest that impacts of curcumin on insulin signaling may be dependent on curcumin concentration, cell types, or physiological and pathophysiological conditions of targeted cells. Although curcumin has been reported to inhibit high glucose-induced proliferation of human retinal endothelial cell (Premanand et al., 2006) and also display beneficial impacts on diabetes-induced endothelial dysfunction (Patumraj et al., 2006; Rungseesantivanon et al., 2010; Nabavi et al., 2015), the potential impacts of curcumin on insulin resistance of vascular endothelial cells and its underlying mechanism(s) remain poorly understood.

The article "Curcumin Improves Palmitate-Induced Insulin Resistance in Human Umbilical Vein Endothelial Cells by Maintaining Proteostasis in Endoplasmic Reticulum" was retracted in 2023. Reasons: original data or images not available; unreliable data; unreliable results or conclusions; concerns about the images.

Endoplasmic reticulum (ER) is one of the major sites for synthesis, folding, maturation, and translocation of most intracellular protein. Protein synthesis and folding processes can lead to accumulation of unfolded or misfolded proteins in the ER lumen, and thus initiate proteolytic mechanisms to remove unfolded or misfolded proteins, as well as aggregated proteins. The process of degradation and clearance of proteins from the ER system is called ER-associated degradation (ERAD), including ubiquitin/proteasome ERAD (I) and autophagy/lysosomal ERAD (II) (Fujita et al., 2007; Kondratyev et al., 2007). If unfolded or aggregated proteins are largely accumulated in the ER lumen, an adaptation program known as unfolded protein response (UPR) will be triggered to increase the ability of ER to fold and degrade proteins. Long-term or inappropriate UPR has a direct causal relationship with insulin resistance (Marciniak and Ron, 2006; Hotamisligil, 2010). Previous studies have shown a significant association between ER stress and insulin resistance in endothelial cells (Lenna et al., 2014; Gustavo Vazquez-Jimenez et al., 2016).When this ER stress is blocked pharmacologically, a complete recovery of insulin sensitivity is achieved (Ozcan et al., 2004). Interestingly, curcumin acts as an inhibitor of both proteasome and ER stress (Milacic et al., 2008; Han et al., 2012; Afrin et al., 2015; Chen et al., 2015; Rashid and Sil, 2015; Wang et al., 2016). Given that the proteasome pathway and autophagy has been demonstrated to interact each other (Korolchuk et al., 2009; Jänen et al., 2010; Wang and Wang, 2015), we rationally and logically speculated that curcumin might maintain ER proteostasis through activating autophagy, leading to suppression of ER stress with subsequent improvement of insulin sensitivity. This hypothesis would be studied in human umbilical vein endothelial cells (HUVECs) treated with saturated fatty acid palmitate.

## Materials and Methods

### Antibodies and Reagents

Antibodies to Akt (#9272), GLUT4 (#2231), IRS-1 (#2382), caveolin-1 (#3238), PERK (#3192), eIF2α (#9722), CHOP (#2895), XBP-1s (#12782), and phospho-specific antibodies to Akt Thr308 (#9275), IRS-1 Ser307 (#2381), and eIF2α Ser 51 (#9721) were from Cell Signaling Technology (Beverly, MA, USA). Anti-ubiquitin (ab7780), PERK Thr982 (ab192591), JNK (ab112501), and JNK1 Thr183 (ab47337) antibodies were obtained from Abcam Inc. (Cambridge, MA, USA). Anti-LC3 (M152-3) and Atg5 (M153-3) monoclonal antibodies were purchased from MBL (Nagoya, Japan). Bafilomycin A1 (BFA, B1793) and curcumin (C1386) were from Sigma-Aldrich Corp. (St. Louis, MO, USA). The Fluorometric substrates of proteasome Suc-LLVY-AMC (S-280), Suc-LLE-AMC (S-230), AC-RLR-AMC (S-300) were purchased from Boston Biochem (Cambridge, MA, USA).

The article "Curcumin Improves Palmitate-Induced Insulin Resistance in Human Umbilical Vein Endothelial Cells by Maintaining Proteostasis in Endoplasmic Reticulum" was retracted in 2023. Reasons: original data or images not available; unreliable data; unreliable results or conclusions; concerns about the images.

### Cell Culture and Treatment

Primary HUVECs were purchased from Invitrogen (Carlsbad, CA, USA) and cultured in phenol red-free Medium 200 (Cat. no. M-200-500; Invitrogen) containing 1% low serum growth supplement (LSGS), 100 μg/ml streptomycin, and 100 units/ml penicillin at 37°C and 5% CO_2_. Palmitate acid (P0500, Sigma-Aldrich, St. Louis, MO, USA) was dissolved in ethanol, mixed with 20% of free fatty acid (FFA)-free BSA, and then incubated overnight at 4°C. Insulin resistance was induced as previously described (Gustavo Vazquez-Jimenez et al., 2016). Briefly, HUVECs were plated in 6-well plates or 60 mm dishes until cells have reached 80% confluence and then incubated with serum-free Medium 200 for another 6 h before palmitate supplementation. After treatment with palmitate, cells were stimulated with 100 nM insulin for 10 min. The same concentration of ethanol mixed with 20% of FFA-free BSA was served as control.

### Glucose Uptake

Glucose uptake was determined using Glucose Uptake Colorimetric Assay Kit (ab136955, Abcam, Cambridge, MA, USA) according to the manufacturer’s instruction. Measurements were performed at least three replicates and then averaged.

### Preparation of Plasma Membrane

Plasma Membrane Protein Extraction Kit (Abcam, Cambridge, MA, USA) was used to obtain plasma membrane (PM) fraction from the cells, according to the manufacturer’s protocol. PM purity was determined by expression of membrane marker caveolin-1.

### Small Interfering RNAs (siRNAs) and Transfection

The siRNA targeting human ATG5 (NM_001286106) was synthesized by QIAGEN China (Shanghai) Co., Ltd (Shanghai, China). The most effective sequences of siRNA and its paired control used in the experiments were as follows: ATG5, 5′-AACACCTCTGCAGTGGCTGAGTGAA-3′, scramble control, 5′-AACTCTCGACGCGGTGAGTTCAGAA-3′. Transfection was performed with 120 pM of siRNA using Lipofectamine^®^ RNAiMAX Transfection Reagent (Invitrogen, Carlsbad, CA, USA) according to the manufacturer’s protocol. The knockdown efficiency was assessed by western blot.

### Peptidase Activity Assays

Proteasomal peptidase activities in HUVECs were measured as described previously (Naujokat et al., 2007; Zhang et al., 2015). Briefly, the lysate was obtained using cytosolic extraction buffer (containing 50 mM HEPES, pH 7.5, 20 mM KCl, 5 mM MgCl_2_, 2 mM ATP, 1 mM DTT, 0.025% digitonin) and then centrifuged at 10,000 × *g* for 10 min at 4°C. The supernatants were collected for determination of protein concentration and peptidase activity assays. The synthetic fluorogenic peptide substrates Suc-LLVY-AMC, Suc-LLE-AMC, and AC-RLR-AMC were used for assaying chymotrypsin-, caspase-, and trypsin-like activities of 20S proteasome, respectively. For assay specificity, 1 μM of proteasome inhibitor MG132 was incubated with the extract. After 90 min of incubation at 37°C, the fluorescence intensity was read using fluorescence spectrometer (Perkin Elmer precisely LS 55, Billerica, MA, USA) at an excitation wavelength of 350 nm and emission wavelength of 440 nm.

The article "Curcumin Improves Palmitate-Induced Insulin Resistance in Human Umbilical Vein Endothelial Cells by Maintaining Proteostasis in Endoplasmic Reticulum" was retracted in 2023. Reasons: original data or images not available; unreliable data; unreliable results or conclusions; concerns about the images.

### Western Blot and Protein Aggregation Assay

The cell lysates were extracted by lysis buffer (containing 50 mM HEPES, pH 7.6, 150 mM NaCl, 1% Triton X-100, 10 mM NaF, 20 mM Na_4_P_2_O_7_, 20 mM β-glycerol phosphate, 1 mM Na_3_VO_4_, 10 mg/ml leupeptin, 10 mg/ml aprotinin, and 1 mM PMSF), incubated on ice for 20 min, and then centrifuged at 14000 × *g* for 10 min at 4°C. The supernatants were mixed with equal volume of 2x SDS-PAGE sample loading buffer and then denatured at 100°C for 10 min. The proteins were separated by SDS-PAGE gel, transferred to a nitrocellulose membrane, incubated with specific primary antibodies for overnight, and detected with horseradish peroxidase (HRP)-conjugated secondary antibodies by using a VersaDoc Image System (BioRad, Hercules, CA, USA).

Protein aggregation was determined using ProteoStat^TM^ Protein Aggregation Assay Kit (ENZ-51023-KP002) from Enzo Life Sciences International Inc. (Plymouth Meeting, PA, USA), following the manufacturer’s instruction.

### Statistical Analysis

The data are presented as the means ± SD. The variable is normally distributed and differences between the groups were examined for statistical significance using analysis of variance (ANOVA), followed by a Newman–Keuls *post hoc* test. Differences were considered significant at *p* < 0.05. All experiments were repeated at least four times with similar results. Representative western blot images were shown in Figures.

## Results

### Curcumin Improved Palmitate-Induced Insulin Resistance in HUVECs

To figure out optimal experimental conditions for palmitate-induced insulin resistance, HUVECs were starved serum for 6 h and then treated with 0.25, 0.5, and 0.75 mM palmitate for 12 h, or 0.5 mM palmitate for 6, 12, and 18 h, followed by stimulation with 100 nM insulin for 10 min. We found that palmitate induced insulin resistance in time- and concentration-dependent manners, as demonstrated by decreased insulin-stimulated phosphorylation of Akt at Thr308 (**Figures 1A,B**). Because the reduction of Akt phosphorylation on Thr308 has statistical significance with 0.5 mM palmitate treatment for 12 h, this concentration and treatment duration of palmitate was used for further experimentation.

The article "Curcumin Improves Palmitate-Induced Insulin Resistance in Human Umbilical Vein Endothelial Cells by Maintaining Proteostasis in Endoplasmic Reticulum" was retracted in 2023. Reasons: original data or images not available; unreliable data; unreliable results or conclusions; concerns about the images.

**FIGURE 1:** **Curcumin mitigated palmitate-induced insulin resistance in HUVECs. (A)** Dose-response effect of palmitate (PA) on insulin (INS)-stimulated Akt T308 phosphorylation. **(B)** Time-response effect of PA on insulin-stimulated Akt T308 phosphorylation. **(C)** Attenuation of insulin resistance by curcumin (Cur) administration. **(D)** Effect of Cur on plasma membrane (PM) translocation of GLUT4. **(E)** Effect of Cur on 2-Deoxy-D-glucose (2-DG) uptake. *N* = 4. ^∗^*p* < 0.05, ^∗∗^*p* < 0.01, ^∗∗∗^*p* < 0.001 vs. indicated groups.

When serum-starved HUVECs were treated with 0.5 mM palmitate in the presence or absence of 2.5, 5, 10, and 20 μM curcumin for 12 h, followed by stimulation with or without 100 nM insulin for 10 min, we found that curcumin supplementation significantly reverted insulin-stimulated phosphorylation of Akt Thr308 (**Figure 1C**). Consistent with these results, curcumin administration reversed the detrimental effects of palmitate on insulin-stimulated GLUT4 translocation on PM (**Figure 1D**) and 2-DG uptake (**Figure 1E**) in HUVECs cotreated with 0.5 mM palmitate and 10 μM curcumin under stimulation with 100 nM insulin for 10 min. These findings suggest that curcumin could sensitize insulin signaling in palmitate-treated HUVECs.

### Palmitate Induced ER Stress and Adaptive Activation of the UPS and Autophagy

To elucidate the mechanism underlying palmitate-induced insulin resistance, we observed the potential impacts of palmitate on ER stress, the ubiquitin-proteasome system (UPS), and autophagy. HUVECs were starved serum for 6 h and then treated with 0.5 mM palmitate for 6, 12, and 18 h. As shown in **Figure 2**, palmitate treatment time-dependently increased the levels of ER stress markers (**Figure 2A**), the ratio of LC3-II to LC3-I (**Figure 2B**), and peptidase activities of 20S proteasome (**Figure 2C**), suggesting that palmitate activated ER stress, the UPS, and autophagy.

**FIGURE 2:** **Palmitate enhanced ER stress and activated autophagy and the ubiquitin-proteasome system (UPS) in HUVECs. (A)** Effect of palmitate (PA) on ER stress markers. **(B)** Effect of PA on LC3 levels. **(C)** Effect of PA on peptidase activities of 20S proteasome. *N* = 4. ^∗^*p* < 0.05, ^∗∗^*p* < 0.01 vs. control group.

When serum-starved HUVECs were pretreated with or without 5 mM 4-phenylbutyric acid (PBA), a potent ER stress inhibitor for 1 h and then incubated in the presence or absence of 0.5 mM palmitate for another 12 h, we found that PBA administration dramatically suppressed palmitate-enhanced LC3-II levels (**Figures 3A,B**), the ratio of LC3-II to LC3-I (**Figure 3A**), and peptidase activities of 20S proteasome (**Figure 3D**). PBA treatment also significantly decreased autophagy flux when compared with HUVECs treated with palmitate alone (**Figure 3C**). These results indicate that palmitate-induced activation of the UPS and autophagy were mediated by ER stress.

The article "Curcumin Improves Palmitate-Induced Insulin Resistance in Human Umbilical Vein Endothelial Cells by Maintaining Proteostasis in Endoplasmic Reticulum" was retracted in 2023. Reasons: original data or images not available; unreliable data; unreliable results or conclusions; concerns about the images.

**FIGURE 3:** **Inhibition of ER stress mitigated palmitate’s impacts on autophagy and the UPS in HUVECs. (A,B)** Reduction of LC3 levels by ER stress inhibitor 4-phenylbutyrate (PBA). **(C)** Attenuation of autophagy flux by PBA. **(D)** Suppression of peptidase activities of 20S proteasome by PBA. *N* = 4. ^∗^*p* < 0.05, ^∗∗^*p* < 0.01 vs. control group; ^#^*p* < 0.05, ^##^*p* < 0.01, ^$^*p* > 0.05 vs. PA-treated group.

### Curcumin Suppressed Palmitate-Induced ER Stress

To figure out the potential impacts of curcumin treatment alone on HUVECs under normal culture condition, HUVECs were starved serum for 6 h and then treated with or without 10 μM curcumin for another 12 h. We found that curcumin treatment alone did not affect expressions of ER stress markers, protein aggregation, and phosphorylation of JNK Thr183 and IRS-1 Ser307 (**Supplementary Figure S1**), suggesting that curcumin did not affect ER stress in HUVECs under normal culture condition.

When serum-starved HUVECs were treated with or without 0.5 mM palmitate in the presence or absence of 10 μM curcumin for 12 h, we found that curcumin treatment markedly decreased the levels of ER stress markers (**Figure 4A**) as well as protein aggregation (**Figure 4B**), which were enhanced by palmitate treatment alone. Additionally, curcumin supplementation significantly inhibited palmitate-elevated expressions of phosphorylation of IRS-1 at Ser307 and JNK at Thr183 (**Figures 4C,D**), suggesting that curcumin could attenuate palmitate-induced ER stress and its downstream molecular events such as activation of JNK/IRS-1 signaling.

**FIGURE 4:** **Curcumin mitigated palmitate-induced ER stress in HUVECs. (A)** Reduction of ER stress markers by curcumin (Cur). **(B)** Mitigation of protein aggregation by Cur. **(C)** Suppression of phosphorylated IRS-1 S307 and JNK Thr183 by Cur. **(D)** Quantification of phosphorylated IRS-1 and JNK in **(C)**. *N* = 4. ^∗^*p* < 0.05, ^∗∗^*p* < 0.01 vs. control group; ^#^*p* < 0.05 vs. PA-treated group.

### Curcumin Inhibited the UPS and Activated Autophagy in Palmitate-Treated HUVECs

To investigate the potential impacts of curcumin on the UPS and autophagy, the serum-starved HUVECs were treated with or without 0.5 mM palmitate in the presence or absence of 10 μM curcumin for 12 h. As shown in **Figure 5**, curcumin supplementation inhibited the UPS and enhanced autophagy, as evidenced by the suppressed peptidase activities of 20S proteasome (**Figure 5A**), increased LC3 levels and the ratio of LC3-II to LC3-1 (**Figures 5C,D**), as well as increased autophagy flux (**Figure 5E**), when compared with the group treated with palmitate alone. The total protein ubiquitination in curcumin-treated HUVECs had a little bit increase but no statistically significant changes (**Figure 5B**).

The article "Curcumin Improves Palmitate-Induced Insulin Resistance in Human Umbilical Vein Endothelial Cells by Maintaining Proteostasis in Endoplasmic Reticulum" was retracted in 2023. Reasons: original data or images not available; unreliable data; unreliable results or conclusions; concerns about the images.

**FIGURE 5:** **Curcumin inhibited the UPS and activated autophagy in HUVECs. (A)** Inhibition of peptidase activities of 20S proteasome by curcumin (Cur). **(B)** Effect of Cur on total protein ubiquitination. **(C)** Enhancement of LC3 levels by Cur. **(D,E)** Increased autophagy flux by Cur. *N* = 4. ^∗^*p* < 0.05, ^∗∗^*p* < 0.01 vs. control group; ^#^*p* < 0.05, ^##^*p* < 0.01 vs. PA-treated group.

### Inhibition of Autophagy Abolished the Beneficial Effect of Curcumin on Palmiated-Induced Insulin Resistance

To confirm the critical role of autophagy in mediating curcumin action on palmitate-induced insulin resistance, we silenced Atg5, an important regulator of autophagy by siRNA technique. The siRNA- and scramble control-infected HUVECs were starved serum for 6 h and then incubated with or without 0.5 mM palmitate in the presence or absence of 10 μM curcumin for another 12 h. We found that Atg5 knockdown abolished the beneficial effects of curcumin on the levels of ER stress markers (**Figure 6A**), exacerbated total protein ubiquitination (**Figure 6B**), and reversed protein aggregation (**Figure 6C**) under combined treatment with curcumin and palmitate, suggesting that Atg5 knockdown counteracted curcumin action on palmitate-induced ER stress. This conclusion was further confirmed by restored phosphorylation of IRS-1 at Ser307 and JNK at Thr183 in Atg5 knockdown HUVECs cotreated with curcumin and palmitate (**Figures 6D,E**).

**FIGURE 6:** **Inhibition of autophagy abolished curcumin’s impacts on ER stress in HUVECs. (A)** Effect of Atg5 knockdown on ER stress markers. **(B)** Effect of Atg5 knockdown on total protein ubiquitination. **(C)** Effect of Atg5 knockdown on protein aggregation. **(D)** Effect of Atg5 knockdown on phosphorylation of IRS-1 S307 and JNK Thr183. **(E)** Quantification of phosphorylated IRS-1 and JNK in **(D)**. *N* = 4. ^∗^*p* < 0.05, ^∗∗^*p* < 0.01 vs. indicated groups.

We next observed the pathophysiological impacts of Atg5 knockdown on insulin signaling. Atg5 knockdown or scramble control HUVECs were starved serum for 6 h and then incubated with or without 0.5 mM palmitate in the presence or absence of 10 μM curcumin for another 12 h, followed by stimulation with 100 nM insulin for 10 min. As shown in **Figure 7**, Atg5 knockdown inhibited insulin-stimulated Akt-Thr308 phosphorylation (**Figure 7A**), GLUT4 PM translocation (**Figure 7B**), and 2-DG uptake (**Figure 7C**), when compared with group cotreated with curcumin and palmitate.

The article "Curcumin Improves Palmitate-Induced Insulin Resistance in Human Umbilical Vein Endothelial Cells by Maintaining Proteostasis in Endoplasmic Reticulum" was retracted in 2023. Reasons: original data or images not available; unreliable data; unreliable results or conclusions; concerns about the images.

**FIGURE 7:** **Inhibition of autophagy abolished curcumin’s impacts on insulin resistance in HUVECs. (A)** Effect of Atg5 knockdown on insulin (INS)-stimulated Akt phosphorylation at Thr308 residue. **(B)** Effect of Atg5 knockdown on PM translocation of GLUT4. **(C)** Effect of Atg5 knockdown on 2-Deoxy-D-glucose (2-DG) uptake. *N* = 4. ^∗^*p* < 0.05, ^∗∗^*p* < 0.01 vs. indicated groups.

Taken together, these results suggest that autophagy mediated curcumin’s protection against palmitate-induced insulin resistance in HUVECs.

## Discussion

It has been suggested that increased concentration of plasma FFAs is an independent predictor of type 2 diabetes in individuals with impaired glucose tolerance (Ly et al., 2017). As one of most abundant FFAs in plasma, palmitate is closely associated with pathogenesis and progression of insulin resistance in insulin-target tissues and cells through inducing oxidative stress, ER stress, and inflammation (Jung et al., 2015; Ly et al., 2017). The previous studies have also demonstrated the inhibitory impacts of the elevated palmitate concentration on cell function and insulin signaling of endothelial cells (Kim et al., 2005; Lu et al., 2013; Gustavo Vazquez-Jimenez et al., 2016). Consistent with these views, we found that palmitate induced insulin resistance in HUVECs in time- and concentration-dependent manners (**Figures 1A,B**). Moreover, palmitate-induced insulin resistance was accompanied with enhanced ER stress (**Figure 2A**), which has been suggested a major contributor to palmitate-induced insulin resistance through ER stress-activated JNK/IRS-1 pathway (Chan et al., 2013; Simon-Szabó et al., 2014; Tang et al., 2015; Park et al., 2016). Indeed, our results found that palmitate stimulated JNK/IRS-1 pathway (**Figures 4C,D**). Thus, our findings evidenced the involvement of ER stress in palmitate-induced insulin resistance of HUVECs.

Curcumin has been proven to enhance insulin receptor activity, sensitize insulin signaling, and inhibit inflammation and oxidative stress under insulin resistance condition, which are collectively responsible for improvement of insulin resistance by curcumin (Jiménez-Osorio et al., 2016). In addition, curcumin displays a specific ability to ameliorate ER stress (Afrin et al., 2015; Rashid and Sil, 2015; Wang et al., 2016). In the present study, we found that curcumin supplementation significantly mitigated palmitate-induced insulin resistance (**Figures 1C–E**) and suppressed palmitate-stimulated ER stress/JNK/IRS-1 signaling in HUVECs (**Figure 4**), suggesting that curcumin reverted palmitate-induced insulin resistance of HUVECs by inhibiting ER stress.

The article "Curcumin Improves Palmitate-Induced Insulin Resistance in Human Umbilical Vein Endothelial Cells by Maintaining Proteostasis in Endoplasmic Reticulum" was retracted in 2023. Reasons: original data or images not available; unreliable data; unreliable results or conclusions; concerns about the images.

It is well known that protein folding stress in ER may result in activation of ER membrane kinases such as PERK leading to UPR, aimed to maintain ER-derived quality control (ERQC) through activating ubiquitin-proteasome ERAD (I) and autophagy/lysosome ERAD (II) (Fujita et al., 2007; Kondratyev et al., 2007). Consistent with the previous studies showing the effective activation of autophagy and the UPS by palmitate (Weigert et al., 2004; Ishii et al., 2015; Janikiewicz et al., 2015; Park et al., 2015; Liu et al., 2016), we found that palmitate treatment significant increased LC3-II levels and peptidase activities of 20S proteasome (**Figures 2B,C**). However, inhibition of ER stress by its specific inhibitor PBA abolished palmitate-stimulated activation of autophagy and the UPS, as evidenced by significant decreases of the ratio of LC3-II to LC3-I, autophagy flux, and peptidase activities of 20S proteasome (**Figure 3**), suggesting that palmitate-induced activation of autophagy and the UPS is an adaptive response to palmitate-stimulated ER stress (Park et al., 2015).

The impacts of autophagy and the UPS on insulin signaling are complex and contradictory as well. Early studies have suggested that overactivation of either autophagy or the UPS negatively regulates insulin sensitivity (Balasubramanyam et al., 2005; Kovsan et al., 2011; Mellor et al., 2011), through reducing intracellular levels of some important molecules of insulin signaling pathway such as insulin receptor and IRS-1/2 in lysosome- or ubiquitin/proteasome-dependent machinery, respectively (Zhou et al., 2009; Leng et al., 2010; Ishii et al., 2015). However, the accumulating evidence has shown that both autophagy and the UPS are necessary for preserving insulin action. Inadequate autophagy contributes to endothelial dysfunction in patients with diabetes (Fetterman et al., 2016). Upregulation of autophagy has been demonstrated to improve insulin resistance, glucose intolerance, hyperglycemia, hyperlipidemia, and diabetic complications (Fujitani et al., 2009; Codogno and Meijer, 2010; Li and Lerman, 2012; Zhang et al., 2015; Kang et al., 2016). Similarly, proteasome inhibition can significantly impair insulin signaling in 3T3-L1 adipocytes or further exacerbate insulin resistance in the myotubes derived from type 2 diabetic patients (Al-Khalili et al., 2014; Díaz-Ruiz et al., 2015). These findings strongly indicate that autophagy and the UPS may be the targets for therapy of diabetes and diabetic complications. The different results of autophagy and the UPS on insulin signaling maybe caused by or associated with cell types or/and experimental conditions. In the present study, we observed an adaptive activation of autophagy and the UPS by palmitate treatment; however, intracellular abundances of key insulin signaling molecules such as insulin receptor, IRS-1, PDK1, and Akt remained unchanged (Data not shown). Combined with our results showing palmitate-induced insulin resistance (**Figures 1A,B**), our findings indicated that this adaptive regulation of autophagy and the UPS did not, at least in this case, affect insulin signaling.

The article "Curcumin Improves Palmitate-Induced Insulin Resistance in Human Umbilical Vein Endothelial Cells by Maintaining Proteostasis in Endoplasmic Reticulum" was retracted in 2023. Reasons: original data or images not available; unreliable data; unreliable results or conclusions; concerns about the images.

The UPS and autophagy break down unnecessary or dysfunctional intracellular proteins through ubiquitin-proteasomal or lysosomal degradation process, respectively (Wang and Wang, 2015). The UPS impairment or inhibition will result in accumulation of misfolded and aggregated protein leading to compensative activation of autophagy (Korolchuk et al., 2009; Jänen et al., 2010; Wang and Wang, 2015), aimed to clear up the aggregated or misfolded proteins that were previously thought to be targeted exclusively by the UPS (Ding et al., 2007; Graziotto et al., 2012). Curcumin possesses the properties of proteasome inhibitor and autophagy inducer (Milacic et al., 2008; Han et al., 2012; Chen et al., 2015). In the present study, we found that curcumin administration significantly suppressed peptidase activities of 20S proteasome, and compensatively activated autophagy under palmitate treatment (**Figure 5**). Hence, the curcumin-induced inhibition of the UPS function did not significantly increase total protein ubiquitination (**Figure 5B**). In contrast, the compensative activation of autophagy would help to eliminate the aggregated proteins, as evidenced by decreased protein aggregation (**Figure 4B**). As discussed above, the UPS and autophagy play a critical role in maintaining ER protein homeostasis by removing most damaged or unfolded proteins as well as aggregated proteins (Fujita et al., 2007; Kondratyev et al., 2007). Inhibition of the UPS and autophagy will result in ER stress (Cybulsky, 2013; Fan et al., 2016; Li et al., 2016). Given that proteasome inhibition or impairment by curcumin compensatively activated autophagy (**Figure 5**), the curcumin-activated autophagy would therefore bring beneficial effects on protein aggregation and ER stress (**Figures 4A,B**), leading to inhibition of JNK/IRS-1 pathway (**Figures 4C,D**).

It is noteworthy that inhibition of autophagy will compromise the UPS function (Korolchuk et al., 2009; Wang and Wang, 2015), which may cause disturbance of ER proteostasis leading to ER stress. Our previous study on 3T3-L1 adipocytes shows that autophagy inability suppresses proteasome activity, induces ER stress, and results in insulin resistance (Zhang et al., 2015). Moreover, inhibition of the UPS function exacerbates autophagy inhibition-induced ER stress (Zhang et al., 2015). Consistent with this research, we found that autophagy inhibition by silencing Atg5, a key regulatory protein of autophagy, attenuated proteasome activity and enhanced ER/JNK/IRS-1 pathway, leading to insulin resistance in HUVECs under normal culture condition (**Supplementary Figure S2**). In addition, Atg5 knockdown abolished the favorable effects of curcumin on ER stress and JNK/IRS-1 pathway (**Figure 6**). Autophagy inhibition also restored protein aggregation (**Figure 6C**) and exacerbated total protein ubiquitination (**Figure 6B**), collectively responsible for restoration of ER stress by palmitate. As consequent, the curcumin-induced improvement of insulin resistance was abolished by the autophagy inhibition (**Figure 7**). These findings strongly suggest that autophagy plays a pivotal role in mediating curcumin action through maintaining ER proteostasis.

The article "Curcumin Improves Palmitate-Induced Insulin Resistance in Human Umbilical Vein Endothelial Cells by Maintaining Proteostasis in Endoplasmic Reticulum" was retracted in 2023. Reasons: original data or images not available; unreliable data; unreliable results or conclusions; concerns about the images.

Taken together, our results revealed that curcumin heighten autophagy activity that is an essential regulator in the control of ER proteostasis (**Figure 8**). This regulation of ERQC compartment might be the basis of curcumin’s beneficial activities in various pathophysiologic conditions of diabetes and diabetic complications including insulin resistance.

**FIGURE 8:** **A schematic diagram of curcumin’s impact on palmitate-induced insulin resistance of HUVECs**. Palmitate-induced disturbance of ER proteostasis results in ER stress/UPR and the adaptive activation of both the UPS and autophagy (black). The chronic ER stress/UPR leads to insulin resistance. Curcumin administration suppresses the UPS function and greatly activates autophagy, leading to restoration of ER proteostasis, inhibition of ER stress/UPR (red), and subsequent improvement of insulin sensitivity in HUVECs.

### Limitations

In the present study, we found that palmitate-induced insulin resistance was significantly attenuated by curcumin-stimulated compensative activation of autophagy but not by palmitate-induced adaptive activation of autophagy. However, we could not definitely explain mechanism underlying this phenomenon. In addition, ER stress, inflammation, and oxidative stress are all associated with the impacts of palmitate and curcumin on insulin signaling (Jung et al., 2015; Jiménez-Osorio et al., 2016; Ly et al., 2017). Although it is well known that these stress processes are intimately interrelated and affect each other (Zhang et al., 2006; Malhotra and Kaufman, 2007; Han et al., 2013), the mechanisms linking ER stress to oxidative stress and inflammation were not investigated in this study. Not only are future studies required to observe how curcumin affect palmitate-induced inflammation and oxidative, but studies also are required to understand how interactions between ER stress, oxidative stress, and inflammation are involved in curcumin action.

The article "Curcumin Improves Palmitate-Induced Insulin Resistance in Human Umbilical Vein Endothelial Cells by Maintaining Proteostasis in Endoplasmic Reticulum" was retracted in 2023. Reasons: original data or images not available; unreliable data; unreliable results or conclusions; concerns about the images.

## Author Contributions

CW, MY, and HQ designed the studies. MY, HQ, YC, MZ, YM, and JY performed the experiments. CW, MY, and YC conducted statistical analyses. CW wrote the manuscript. All authors approved submission of the manuscript.

## Conflict of Interest Statement

The authors declare that the research was conducted in the absence of any commercial or financial relationships that could be construed as a potential conflict of interest.

## Supplementary Material

FIGURE S1 **Curcumin’s impacts on ER stress in HUVECs under normal culture condition**. HUVECs were starved serum for 6 h and then treated with or without 10 μM curcumin for another 12 h. **(A)** Effects of curcumin on ER stress markers. **(B)** Effects of curcumin on protein aggregation. **(C)** Effect of curcumin on phosphorylation of IRS-1 S307 and JNK Thr183. *N* = 4. ^#^*p* > 0.05 vs. control group.

FIGURE S2 **Atg5 knockdown induced insulin resistance in HUVECs under normal culture condition**. The siRNA- and scramble control-infected HUVECs were starved serum for 6 h and then stimulated with or without 100 nM insulin for 10 min. **(A)** Effects of Atg5 knockdown on chymotrypsin peptidase activities of 20S proteasome. **(B)** Effects of Atg5 knockdown on ER stress markers. **(C)** Effect of Atg5 knockdown on phosphorylation of IRS-1 S307 and JNK Thr183. **(D)** Effect of Atg5 knockdown on insulin (INS)-stimulated Akt phosphorylation at Thr308 residue. **(E)** Effect of Atg5 knockdown on 2-Deoxy-D-glucose (2-DG) uptake. *N* = 4. ^∗∗^*p* < 0.01, ^∗∗∗^*p* < 0.001 vs. scramble control or indicated groups.
